This article has been retracted.

# Improved Outside-In Suture through the Joint Capsule to Repair the Palmer I-B Triangular Fibrocartilage Complex Superficial Injury

**DOI:** 10.1155/2021/8387813

**Published:** 2021-11-10

**Authors:** Tonglong Xu, Xiaoyun Pan, Jingyi Mi

**Affiliations:** ^1^Medical College, Soochow University, Suzhou, China; ^2^Wuxi 9th People's Hospital Affiliated to Soochow University, Liangxi Road, No.999, Binhu District, Wuxi, Jiangsu, China

## Abstract

**Background:**

The treatment of type I-B triangular fibrocartilage complex superficial injury is always a challenge to orthopedists. The traditional outside-in suture method often causes a risk of nervous irritation. We designed a modified outside-in suture through the joint capsule to repair the Palmer I-B triangular fibrocartilage complex superficial injury.

**Methods:**

From December 2014 to December 2018, we retrospectively collected the medical records of 18 patients in our hospital who used the modified outside-in suture through the joint capsule to repair type I-B triangular fibrocartilage complex superficial injury. Among them, there were 12 males and 6 females, with an average age of 36.2 years. There were 6 cases on the left side and 12 cases on the right side. Record the healing time of all patients after surgery and the occurrence of related complications, and record the pain visual analogue scale (VAS), grip strength, wrist flexion and extension, radioulnar deviation and forearm rotation range of motion, modified Mayo wrist joint function score, and disability of arm-shoulder-hand (DASH) score before operation and at the last follow-up.

**Results:**

One patient was lost to follow-up, and a total of 17 patients received the final follow-up. Patients were followed up for 24 to 36 months, with an average of 29.6 ± 3.0 months. No wound infection, nerve damage, or irritation occurred after the operation. At the last follow-up, 15 cases of wrist pain disappeared completely, and 2 cases had mild discomfort during exercise. At the last follow-up, VAS decreased from 3.8 ± 0.7 points before operation to 0.8 ± 0.7 points (*P* < 0.05); grip strength increased from 15.1 ± 3.1 kg before operation to 23.2 ± 1.5 kg (*P* < 0.05); wrist flexion and extension, radioulnar deflection, and forearm rotational mobility increased from 116.3 ± 2.2°, 37.0 ± 3.5°, and 141.6 ± 2.2° before operation to 117.2 ± 2.5° (*P* < 0.05), 38.9 ± 3.0° (*P* < 0.05), and 142.4 ± 1.9° (*P* < 0.05), respectively; the modified Mayo wrist joint function score increased from 66.1 ± 3.6 points to 82.5 ± 3.9 points (*P* < 0.05), of which 10 cases were excellent, 5 cases were good, 2 cases were fair, and the excellent and good rate was 88.2%; DASH score improved from 37.0 ± 5.7 points preoperatively to 8.0 ± 2.5 points (*P* < 0.05).

**Conclusion:**

The modified outside-in suture through the joint capsule to repair the superficial injury of Palmer I-B triangular fibrocartilage complex has a good clinical effect and is worthy of clinical widespread promotion.

## 1. Introduction

In recent years, with the popularity of national sports, sports-related injuries have become more and more common. When the wrist is supported on the ground during a fall or suffered violent swing movement, some patients often experience varying degrees of pain and discomfort in the wrist joints. If the pain appears on the ulnar side, it is likely that a triangular fibrocartilage complex (TFCC) injury has occurred. This injury is the main cause of wrist ulnar pain, and it is also a major research hotspot in the field of wrist joints. Palmer I-B injury is the most common type of injury in clinical practice [1]. For patients with I-B injuries who have failed conservative treatment or have surgical indications, surgery is generally required. According to different types of injury, such as simple superficial ligament injury or combined deep ligament injury, the current surgical methods mainly include transarticular capsule repair, ulnar foveal ligament stop point reconstruction, ligament transplantation reconstruction, and distal radioulnar joint replacement or plastic surgery [2–17]. For patients with simple superficial ligament injury, the current mainstream repair method is the outside-in suture through the joint capsule [2, 3, 11, 17]. However, many scholars have reported that patients treated by outside-in suture method have found that the dorsal branch of the ulnar nerve is injured or the local irritation symptoms are found. This is often caused by the suture knot irritating the dorsal branch of the ulnar nerve or the skin [2, 3, 11, 17]. Our research group innovatively modified the traditional outside-in suture of the joint capsule and modified the traditional extracapsular suture to intracapsular suture and found that the incidence of postoperative nerve irritation in patients can be significantly reduced. From December 2014 to December 2018, we retrospectively collected the medical records of 18 patients in our hospital who used the modified outside-in suture through the joint capsule to repair the Palmer I-B TFCC superficial injury. The analysis found that the patients were satisfied with the curative effect and it is worthy of clinical promotion.

## 2. Materials and Methods

### 2.1. General Materials

The inclusion criteria were as follows: (1) unilateral Palmer I-B TFCC superficial injury; (2) normally healthy, no other diseases; (3) failed conservative treatment for more than 3 months; and (4) no history of trauma to the wrist. The exclusion criteria were as follows: (1) combined with other injuries; (2) obvious instability of the lower radioulnar joint; (3) without conservative treatment for more than 3 months; (4) open injuries or complications such as fractures and vascular and nerve injuries.

From December 2014 to December 2018, according to the inclusion and exclusion criteria, a total of 18 patients in our hospital who used the modified outside-in suture through the joint capsule to repair Palmer I-B TFCC superficial injury were collected. Among them, there were 12 males and 6 females, with an average age of 36.2 years. There were 6 cases on the left side and 12 cases on the right side. Record the healing time of all patients after surgery and the occurrence of related complications, and record the VAS of pain, grip strength, wrist flexion and extension, radioulnar deviation and forearm rotation range of motion, modified Mayo wrist Joint function score, and DASH score before operation and at the last follow-up.

### 2.2. Surgical Methods

The patient was placed in the supine position, and routinely used brachial plexus block anesthesia was administered. The airbag tourniquet on the upper arm was set up at 36 kPa, upper limb abduction and elbow were fixed at 90° position, and middle and ring fingers were tracked and fixed on the Linvatec traction frame with a special mesh finger cuff. The traction force is about 5 kg. The gravity perfusion system is infused with physiological saline. A wrist arthroscopy with a diameter of 2.7 mm and a tilt angle of 30° and a camera (Arthrex, U.S.) and shaver system (Arthrex, U.S.) are used. The arthroscopy is placed in the conventional 3-4 approach, the 4-5 approach is the operating approach, and the 6U approach is generally the water outlet channel. A probe is used to detect intra-articular synovial hyperplasia, TFCC ulnar tear, and whether the TFCC trampoline test is positive. First, clean the proliferative synovium and inflammatory tissue; then, make a longitudinal incision at the 6U approach to expose the joint capsule. The 9-gauge needle and the 12-gauge needle are used to penetrate vertically. After passing the TFCC, use the outside-in suture technique to pass the 2-0 PDS suture through the TFCC and then withdraw it through the connective tissue in the joint capsule, tighten the knot on the inside of the joint capsule, and then use a similar method to pass through the second stitch for reinforcement. Close the joint capsule with continuous sutures. Remove the traction device, check the stability of the DRUJ, loosen the withers, use electrocoagulation hemostasis to stop bleeding, rinse and stitch the wound (Figure 1).

### 2.3. Postoperative Rehabilitation and Efficacy Evaluation

Postoperatively, the elbow joint was fixed at 80° elbow flexion with a long-arm plaster cast, the forearm was in a neutral position, and the wrist was in a neutral position. At 4 weeks after the operation, the plaster was removed and the active and passive extension and flexion of the wrist and fingers and the functional exercise of pronation and supination were started. At 6 weeks after the operation, the weight-bearing activities such as twisting towels and lifting objects were allowed to begin. The patients were followed up regularly in the 2 weeks, 6 weeks, 3 months, and 6 months after the operation and every six months thereafter. MRI examination recorded the healing of the ligament 6 months after the operation. Record the healing time of all patients after surgery and the occurrence of related complications, and record the visual analogue scale (VAS) of pain, grip strength, wrist flexion and extension, radioulnar deviation and forearm rotation range of motion, modified Mayo wrist joint function score, and DASH score before surgery and at the last follow-up.

### 2.4. Data Processing and Statistical Analysis

Use SPSS 23.0 statistical software package (SPSS Inc. Chicago, IL) for statistical analysis. Data are expressed as mean ± standard deviation. Data are compared by paired *t*-test. *P* < 0.05 indicates that the difference is statistically significant.

## 3. Results

One patient was lost to follow-up, and a total of 17 patients received the final follow-up. Patients were followed up for 24 to 36 months, with an average of 29.6 ± 3.0 months. No wound infection, nerve damage, or irritation occurred after the operation. At the last follow-up, 15 cases of wrist pain disappeared completely, and 2 cases had mild discomfort during exercise. At the last follow-up, VAS decreased from 3.8 ± 0.7 points before operation to 0.8 ± 0.7 points (*P* < 0.05); grip strength increased from 15.1 ± 3.1 kg before operation to 23.2 ± 1.5 kg (*P* < 0.05); wrist flexion and extension, radioulnar deflection, and forearm rotational mobility increased from 116.3 ± 2.2°, 37.0 ± 3.5°, and 141.6 ± 2.2° before operation to 117.2 ± 2.5° (*P* < 0.05), 38.9 ± 3.0° (*P* < 0.05), and 142.4 ± 1.9° (*P* < 0.05), respectively; modified Mayo wrist joint function score increased from 66.1 ± 3.6 points to 82.5 ± 3.9 points (*P* < 0.05), of which 10 cases were excellent, 5 cases were good, 2 cases were fair, and the excellent and good rate was 88.2%; DASH score improved from 37.0 ± 5.7 points preoperatively to 8.0 ± 2.5 points (*P* < 0.05) (Table 1).

## 4. Discussion

In our study, the functional scores of 17 patients who received the final follow-up were significantly improved compared with preoperative scores, and none of the 17 patients developed nervous irritation symptoms after operation. This is mainly due to our improvement of the traditional outside-in suture method through the joint capsule. In traditional outside-in suture of the joint capsule, the suture knots are tied on the outside of the joint capsule, and the direction of the dorsal branch of the ulnar nerve is just outside the ulnar joint capsule of the wrist joint and is often located next to the knot. Even if we have avoided the nerve knot during the operation, when the wrist joint is pronated and supinated after the operation, the knot is accompanied by joint rotation, which may still irritate the dorsal branch of the ulnar nerve or cause local skin irritation. Our improved method is to tie a knot inside the joint capsule, thereby effectively isolating the knot from the dorsal branch of the ulnar nerve through the joint capsule, which greatly reduces the possibility of ulnar nerve irritation.

At present, the treatment of Palmer I-B triangular fibrocartilage complex superficial injury through joint capsule suture is the most clinically used operation. Atzei and Luchetti [17] proposed that for Palmer I-B triangular fibrocartilage complex superficial injury, suture through the joint capsule can achieve good results. Soreide et al. [18] followed up 11 patients who underwent outside-in suture through the joint capsule to repair TFCC injuries for up to 20 years and found that most patients achieved satisfactory results. Scholars have also made some explorations on stitching methods. Bayoumy et al. [11] proposed that the horizontal mattress suture is more biomechanically stable than the longitudinal mattress suture and can effectively reduce the cutting effect of the suture, but it still cannot avoid the complications of the ulnar nerve and the irritation of the knot on the skin. Scholars continue to report that patients who repaired the Palmer I-B TFCC superficial injury via joint capsule suture under arthroscopy were found to have symptoms of nerve irritation after surgery [19–20].

Conca et al. [2] proposed that the most commonly used arthroscopic technique for repairing torn TFCC is to repair the superficial ligament with the ulnar joint capsule through the suture of the joint capsular suture technique to restore the tension of the superficial ligament of TFCC and improve the patient's clinical symptoms. However, we all know that patients with Palmer I-B TFCC superficial injury often have no instability or only mild instability in the distal radioulnar joint. Therefore, even if the joint capsule is not sutured in, the stability of patient's distal radioulnar joint is still reliable after surgery, which can be verified by arthroscopic exploration and immediate postoperative impact palpation after we suture. After the modified operation is completed, we can see the tension of the superficial ligament of TFCC restored under arthroscopy, and the trampoline test turns from positive to negative. The impact palpation experiment can verify the stability of the distal radioulnar joint.

However, there are still some shortcomings in this study, with the hope of subsequent improvement: (1) this study is a retrospective study, with low level of evidence, and prospective studies can be designed in the later period; (2) the follow-up time is short, and the early and midterm clinical efficacy is mainly reported at present. We will continue to follow up these patients.

## 5. Conclusion

The modified outside-in suture through the joint capsule has a good midterm clinical effect for repairing Palmer I-B TFCC superficial injury, and it is worthy of widespread clinical application.

## Figures and Tables

**Figure 1:** (a) Tie the knot inside of the joint capsule; (b)close the joint capsule and cover the knots, and continue sutures to reduce the nerve irritation of the knots; (c) verify the stability of the distal radioulnar joint.

**Table 1:** Results before operation and at last follow-up.

	Before operation	Last follow-up	*P* value
VAS	3.8 ± 0.7	0.8 ± 0.7	≤0.001
Grip strength (kg)	15.1 ± 3.1	23.2 ± 1.5	≤0.001
Wrist flexion and extension mobility	116.3 ± 2.2	117.2 ± 2.5	0.001
Wrist radioulnar deflection mobility	37.0 ± 3.5	38.9 ± 3.0	≤0.001
Forearm rotational mobility	141.6 ± 2.2	142.4 ± 1.9	0.011
Modified Mayo wrist joint function	66.1 ± 3.6	82.5 ± 3.9	≤0.001
DASH	37.0 ± 5.7	8.0 ± 2.5	≤0.001

## Data Availability

The data used to support this study are available from the corresponding author upon request.
